# Hip and Knee Joint Angles Determine Fatigue Onset during Quadriceps Neuromuscular Electrical Stimulation

**DOI:** 10.1155/2022/4612867

**Published:** 2022-07-22

**Authors:** Jonathan Galvão Tenório Cavalcante, Álvaro de Almeida Ventura, Leandro Gomes de Jesus Ferreira, Alessandra Martins Melo de Sousa, Ivo Vieira de Sousa Neto, Rita de Cássia Marqueti, Nicolas Babault, João Luiz Quagliotti Durigan

**Affiliations:** ^1^Graduate Program of Rehabilitation Sciences, University of Brasília, Distrito Federal, Brazil; ^2^Graduate Program of Physical Education, University of Brasília, Distrito Federal, Brazil; ^3^Undergraduate Program of Physical Therapy from University of Brasília, Distrito Federal, Brazil; ^4^Graduate Program of Sciences and Technology of Health, University of Brasília, Distrito Federal, Brazil; ^5^Centre d'Expertise de la Performance, INSERM UMR1093-CAPS, University of Burgundy Franche-Comté, UFR des Sciences du Sport, F-21000 Dijon, France

## Abstract

Neuromuscular electrical stimulation (NMES) has been used to increase muscle strength and physical function. However, NMES induces rapid fatigue, limiting its application. To date, the effect of quadriceps femoris (QF) muscle length by knee and hip joint manipulation on NMES-induced contraction fatigability is not clear. We aimed to quantify the effects of different muscle lengths on NMES-induced contraction fatigability, fatigue index, and electromyographic (EMG) activity for QF muscle. QF maximum evoked contraction (QMEC) was applied in a 26 min protocol (10 s on; 120 s off; 12 contractions) in 20 healthy participants (24.0 ± 4.6 years old), over 4 sessions on different days to test different conditions. The tested conditions were as follows: supine with knee flexion of 60° (SUP60), seated with knee flexion of 60° (SIT60), supine with knee flexion of 20° (SUP20), and seated with knee flexion of 20° (SIT20). Contraction fatigability (torque decline assessed by maximal voluntary contraction [MVC] and during NMES), fatigue index (percentage reduction in MVC), and EMG activity (root mean square [RMS] and median frequency) of the superficial QF' constituents were assessed. After NMES, all positions except SUP20 had an absolute reduction in MVC (*p* < .001). Fatigue index was greater in SIT20 than in SIT60 (*p* < .001) and SUP20 (*p* = .01). There was significant torque reduction across the 12 QMEC in SUP60 and SIT60, up to 10.5% (*p* < .001–.005) and 9.49% (*p* < .001–.033), respectively. There was no torque reduction during NMES in SUP20 and SIT20. Fatigue was accompanied by an increase in RMS (*p* = .032) and a decrease in median frequency for SUP60 (*p* < .001). Median frequency increased only in the SUP20 condition (*p* = .021). We concluded that QF NMES-induced contraction fatigability is greater when the knee is flexed at 60° compared to 20°. In addition, a supine position promotes earlier fatigue for a 60° knee flexion, but it delays fatigue onset for a 20° knee flexion compared to the seated position. These results provide a rationale for lower limb positioning during NMES, which depends on training objectives, e.g., strengthening or task-specific functionality training.

## 1. Introduction

Neuromuscular electrical stimulation (NMES) is commonly applied to recover functionality and for muscle strengthening [1, 2]. However, NMES-evoked contractions are more fatiguing and damaging than voluntary contractions, which may limit their applicability [3–5]. Muscle fatigue is a complex and multifactorial phenomenon dependent on changes at both central and peripheral levels [6]. Declines in contraction force induced by NMES are types of performance fatigability (i.e., decrease in an objective measure of performance over a discrete period of time) [7] that hereafter in this manuscript was referred to as “contraction fatigability” or simply “fatigability” [8]. Previous studies have shown the dependency of fatigue onset on muscle length by manipulating joint angle. During fatiguing protocols with voluntary contraction, the dependency of fatigue onset on muscle length by manipulating joint angle has been demonstrated. In extended knee angles, the quadriceps femoris muscle (QF) is less fatigable than in more flexed angles [9, 10], which is regarded to be a consequence of increased metabolism when a greater force is generated, according to the number of actin-myosin cross-bridge interactions [11]. In acknowledging this, manipulating joint angles might also have important implications for balancing force output and fatigability in the NMES isometric protocols.

A previous study showed that QF NMES is more fatiguing at 90° of knee flexion than at 15° (0° is full extension), i.e., at longer muscle length [12]. Another study showed earlier and greater fatigue at 65° compared to 90° or 20° [13], i.e., at a midmuscle length. Increased contraction fatigability in these examples was explained by the greater absolute knee extensor torque in fresh condition. Some elegant studies reported a greater evoked torque in supine (hip extended) compared to seated (hip flexed), which was attributed to an improved length-tension relationship of the rectus femoris (RF) and the biarticular constituent of the QF [14, 15]. However, the influence of muscle length changes, by hip angle manipulation, on NMES-induced contraction fatigability was not investigated to date.

NMES allows the observation of peripheral fatigue onset, i.e., failure in excitation-contraction coupling [16], described as a reduction in force generation capacity without the requirement of voluntary/central command [6]. Moreover, acute changes in maximum voluntary contraction (MVC), accompanied by electromyographic (EMG) signals, may inform how the QF is affected by NMES. EMG has been widely used in muscle fatigue evaluation due to its noninvasiveness, real-time, and applicability. Among the physiological parameters for contraction fatigability assessment [17], root mean square (RMS), a measure of motor unit recruitment [18], and the median frequency, which measures the motor units' firing rate [19] are commonly used. However, these EMG's outcomes were not assessed under the influence of QF muscle length before and after a set of QF maximal evoked contractions (QMEC). Relative changes in spectral parameters of the EMG signals may reflect the intermuscular differences in the synergistic QF constituents [20, 21] and impact the adaptations to NMES training. Moreover, once all QF constituents work as a whole and are interconnected [22, 23], it is possible that by changing the RF length, all the other constituents may display fatigue-related changes.

NMES-induced contraction fatigability could indicate muscle overload, which is desirable for strengthening purposes, but it can also limit a lengthy functional activity duration of a rehabilitative protocol. A detailed understanding of QF fatigability may help in the lower limb position adjustments for NMES isometric protocols. Therefore, we aimed to investigate the effects of different muscle lengths, by changing hip and knee joint angles, on NMES-induced contraction fatigability, fatigue index, and EMG activity of the QF (RF, vastus lateralis [VL], and vastus medialis [VM]). Based on the compelling evidence, we hypothesized that the fatigue would be earlier and greater at muscle lengths at which greater torque is produced.

## 2. Material and Methods

### 2.1. Trial Design and Participants

This was a secondary outcome of a study registered at http://clinicaltrials.gov (NCT03822221). This was a randomized within-subject repeated measure design with the participation of 20 men (mean ± SD) age: 24.0 ± 4.6 (years old), bodyweight: 77.0 ± 9.3 (kg), and height: 177.6 ± 6.3 (cm). All participants were informed about the procedures, benefits, and potential risks and gave written consent to participate. The Research Ethics Committee of the Faculdade de Ceilândia/Universidade de Brasília approved the study (94388718.8.0000.8093) in accordance with the Helsinki Declaration of 1975. The procedures were performed at the Strength Laboratory of the Faculdade de Educação Física/Universidade de Brasília. The manuscript is reported according to the CONSORT (Schulz et al. 2010).

Participants were recruited through flyers distributed at the local university and verbal invitations. The eligibility criteria were 18 to 30 years old, male, healthy, physically active according to the International Physical Activity Questionnaire, and not engaged in systematic strength training of the lower limbs. The exclusion criteria were nonresponsive or important discomfort during NMES (torque < 40% of the MVC for each position), neuromuscular diseases, or musculoskeletal conditions that could limit the experimental procedure.

### 2.2. Randomization and Allocation Concealment

The participants opened an opaque envelope containing four small paper sheets, each drawing and describing a position. They removed each sheet without looking inside the envelope, and the order was registered and used as the sequence of testing. The positions were supine (0° = hip extended) with knee flexion of 60° (0° = full knee extension) (SUP60); seated (hip flexion of 85°) with knee flexion of 60° (SIT60); supine with knee flexion of 20° (SUP20), and seated with knee flexion of 20° (SIT20). These combinations of joint angles were chosen because (1) 60° of knee flexion (or close) is optimal for maximal force generation [24]; (2) it is claimed that QF NMES when the knee is fully extended is practical because it would not be necessary to fix the foot in a specific angle, but this approach may compromise strength gains [25]. Once torque reading in the dynamometer is compromised when the knee is fully extended, we choose 20° of knee flexion to contrast the optimal position while maintaining a short muscle length, commonly 30° or below [26]; (3) QF NMES is commonly applied when the subject is seated, supine, or in between; thus, we chose two far apart positions (0° and 85°) without compromising safety of biomechanics (e.g., hyperextension or leaning forward).

### 2.3. Interventions

This study involved five laboratory visits: a familiarization session and four experimental sessions, each for a position (as described in the randomization). All the sessions were seven days apart, 2-3 hours long, and conducted in the daytime (between 09.00 am and 04.00 pm). Participants were instructed not to ingest alcohol or stimulants (e.g., caffeine, chocolate, and performance supplements), respectively, 24 and 6 hours before visits, to avoid strenuous exercise 36 h before the next session, and to maintain their regular diet.

### 2.4. General Setup

Participants underwent the experiment while positioned on a dynamometer (System 4, Biodex Medical Systems, New York, USA) to measure the extensor torque (voluntary or evoked) of the right knee. The equipment axis was visually aligned with the knee flexion-extension axis, i.e., the lateral epicondyle of the femur. Knee and hip angles were adjusted with a goniometer, and the lever arm of the dynamometer transducer was firmly attached 2-3 cm above the lateral malleolus with a strap. Subjects were firmly stabilized to the chair with belts across the chest and pelvic girdle to minimize body movements.

The EMG of the VL, VM, and RF were recorded bipolarly using three pairs of circular silver chloride electrodes (Ag/Cl), each measuring 20 mm in diameter, with a recording diameter of 10 mm, and separated by an interelectrode distance (center to center) of 20 mm. Each electrode pair was positioned longitudinally on the belly of each superficial muscle of the QF. A reference electrode was fixed on the patella of the ipsilateral lower limb. Prior to electrode placement, trichotomy and cleaning with alcohol were made to reduce the skin impedance (<5 k*Ω*). EMG signals were amplified with a bandwidth frequency between 15 Hz and 500 Hz (common − mode rejection rate = 90 dB; impedance = 100 M*Ω*, gain = 1,000). Then, the root mean square (RMS; in *μ*V) and the median frequency (in Hz) were obtained using the Miotool system (Miotec®) by selecting a 500 ms window in the plateau of the MVC.

### 2.5. Familiarization

Firstly, anthropometric assessment (body mass and height) and motor point localization were performed. Each motor point on the VL and the VM muscles (Botter et al. 2011) was recorded as the distance from the patellar base and the thigh midline to be reproduced in the following sessions. Subsequently, three MVC and three QMEC were performed in each position to familiarize the participants with the procedures and verify responsiveness and comfort during NMES. During each MVC, participants were encouraged verbally to perform maximally and received visual feedback on the torque produced. To achieve the QMEC, the current amplitude was gradually increased in steps of two to 10 mA, according to the participant tolerance. At the same time, participants informed their discomfort using a 0–10 numeric scale after each NMES train, where 0 represented no discomfort and 10 represented the maximal perceived discomfort. Participants were informed that a report of 8 out of 10 of perceived discomfort should correspond to the maximum tolerated current amplitude they were willing to tolerate. Moreover, trials at a given angle would end any time they wished to stop the testing [27]. The maximum current amplitude for each position was registered and used in the subsequent sessions to allow rapid achievement of the QMEC for the fatigue protocol.

### 2.6. Contraction Fatigability Protocol

In each experimental session, one of four positions (SUP60, SIT60, SUP20, and SIT20) was tested for fatigue of the knee extensor QF during and right after a 12-QMEC protocol. Prior to the fatiguing protocol, the participants performed two MVCs while torque and EMG were monitored. The NMES stimulator device (Neurodyn 2.0, Ibramed, SP, Brazil) was connected to two isolated cables, and a pair of self-adhesive electrodes of 25 cm^2^ applied over the motor points. It was used a pulsed current (frequency: 100 Hz, phase duration: 500 *μ*s, rise time: 3 s, on time: 4 s, decay time: 3 s, off time: 2 min). The protocol lasted 26 minutes (12 contractions in total). This was the number of contractions needed for a complete QF imaging assessment during QMEC in a previous study [28]. Volunteers reported discomfort after each QMEC, and the current amplitude was increased (2-5 mA), if necessary, to maintain the target level of discomfort of 8 out of 10, as described in familiarization. Subjects were instructed to fully relax during NMES. All physical parameters of the stimulator were checked using a digital oscilloscope (Model DS1050E; Rigol, Cleveland, Ohio).

### 2.7. Outcomes

Our outcomes were the absolute evoked torque variation across the 12 QMEC and the variation in MVC (absolute and relative) and EMG (RMS and median frequency) before (baseline) and after the fatiguing procedure.

#### 2.7.1. Torque Measurement

Torque recording was performed during the 12 QMEC protocol and the pre- and post-NMES MVC. For the MVC, we used the mean of two attempts separated by 2 min. For both MVC and QMEC and MVC, resting torque was recorded in each position and used for subsequent gravity correction due to the weight of the limb or other force, such as the passive tension of the structures that cross the knee. The torque recording was saved in a computer for subsequent assessment using the data acquisition device New Miotool (Miotec Biomedical Equipment Ltd., POA, Brazil) as an interface with the dynamometer. The data was read in the software MiotecSuite 1.0 (Miotec Equipamentos Biomédicos, RS, Brazil) by selecting a 500 ms window in the peak plateau of each torque.

#### 2.7.2. Contraction Fatigue on Maximal Voluntary Contraction

Contraction fatigability was quantified as the absolute and percentage change between the MVC torque generated pre- (baseline) and post-NMES. The fatigue index was obtained according to the equation: [(post‐NMES MVC–baseline MVC)/post‐NMES MVC] × 100 [29].

#### 2.7.3. Contraction Fatigability Assessment during QMEC

For the fatigue obtained during NMES, contraction fatigability was quantified as the absolute difference between the torque generated during the first QMEC and the following QMECs (12 in total).

#### 2.7.4. Fatigue Assessment from EMG

For the RMS, we showed the raw values (rRMS) of the superficial QF's constituents separately and collapsed (i.e. the mean). Besides, we demonstrated the RMS by summing all constituents and normalizing them by the MVC torque (QF nRMS). This procedure was required to compare conditions with different torques values, once we could not infer the individual contribution to torque of each constituent. Thus, once the QF constituents act in synergy, the effect of the summed RMS from the superficial constituents normalized by the MVC served as a surrogate of the overall activation on the muscle group.

### 2.8. Statistical Analysis

The sample size (*n* = 20) was determined a priori using G∗Power (version 3.1.3; University of Trier, Trier, Germany) with the level of significance set at *p* = 0.05 and power (1 − *β*) = 0.80. All outcomes are reported as mean and its 95% confidence interval (95% CI). A two-way ANOVA (*position* [SUP60, SIT60, SUP20, and SIT20] by *time* [pre- and post-QMEC]) was used to observe differences in MVC and QF nRMS. The contraction fatigability index was analyzed with a one-way ANOVA with a main effect of *position*. A two-way ANOVA (*position* by *time* [from the 1st to the 12th QMEC]) was used to observe differences in evoked torque. A three-way ANOVA (*position* by *muscle* [RF, VL, and VM] by *time* [pre- and post-QMEC]) was used to observe differences in rRMS and median frequency. The significance threshold was set at *α* < 0.05. When a significant difference was detected, a Tukey post hoc test was applied to identify the differences. Effect sizes (partial eta squared-*η*_*ρ*_^2^) and statistical power were calculated. All statistical analyses were performed using Statistica 23.0 (STATSOFT Inc., Tulsa, Oklahoma, USA).

## 3. Results

### 3.1. Contraction Fatigability Assessment during QMEC

There was a significant effect of interaction (*position* by *time*) for the QMEC (*F*_33,627_ = 3.23, *p* < 0.001, *η*_*ρ*_^2^: 0.14, power: 1.0). All significant differences are demonstrated in Figure 1(a), while Figure 1(b) shows the percentage change. The post hoc analysis showed that QMEC was greater in SUP60 than in SIT60 (*p* = 0.001) in the 1^st^ evoked contraction. Moreover, SUP60 and SIT60 had greater QMEC than SUP20 and SIT20 in all contractions (*p* < 0.001). Significant torque reduction occurred only in the SUP60 and SIT60. In the SUP60, the significant reduction occurred from the fifth contraction and progressively in the following contractions (*p* < 0.001–0.005), while significant torque reduction occurred from the seventh contraction and progressively in the following contractions in the SIT60 (*p* < 0.001–0.033).

### 3.2. Contraction Fatigability on Voluntary Contraction

A significant effect of interaction between position and time for the MVC was found (*F*_3,57_ = 3.92, *p* = 0.012, *η*_*ρ*_^2^: 0.17, power: 0.80; Figure 2(a)). Both in the baseline and post-NMES, the MVC was greater in the SUP60 and SIT60 than SUP20 and SIT20 (*p* < 0.001). Comparing the two time-points, the post hoc analysis showed that there was a significant decrease in the MVC in the SUP60 (*p* < 0.001), SIT60 (*p* = 0.001), and SIT20 (*p* < 0.001), but not in SUP20 (*p* = 0.11). The fatigue index is represented in Figure 2(b), which shows that considering the percentage change, SIT20 had greater torque reduction than SIT60 (*p* < 0.001) and SUP20 (*p* = 0.011).

### 3.3. Fatigue Assessment from EMG

There was an effect of interaction of *position* by *muscle* by *time* for the rRMS (*F*_6,114_ = 3.44, *p* = 0.003, *η*_*ρ*_^2^: 0.15, power: 0.93). Comparing baseline and post-NMES, the rRMS reduced for the RF in SIT60 (*p* = 0.010) and SIT20 (*p* = 0.043), and for the VM in SIT20 (*p* > 0.001; Figures 3(c)–3(e)). There was also an interaction of *position* by *time* (*F*_3,57_ = 10.72, *p* < 0.001, *η*_*ρ*_^2^: 0.36, power: 0.99), showed as a surrogate of the QF rRMS by collapsing its superficial constituents (Figure 3(a)). There was a significant reduction in rRMS in SUP20 (*p* = 0.020) and SIT20 (*p* < 0.001) after QMECs compared to baseline.

There was also an interaction of *position* by *time* (*F*_3,57_ = 3.98, *p* < 0.019, *η*_*ρ*_^2^: 0.17, power: 0.81) for the QF nRMS (Figure 3(b)). The post hoc analysis showed an increased nRMS in SUP60 after QMECs compared to baseline (*p* = 0.032). Moreover, in both the baseline and after QMECs, the nRMS was lower in SUP60 and SIT60 compared to SUP20 and SIT20 (*p* < 0.001).

There was an effect of interaction for *position* by *muscle* by *time* for the median frequency (*F*_6,114_ = 2.262, *p* = 0.042, *η*_*ρ*_^2^: 0.10, power: 0.77). The median frequency reduced for the RF in SUP60 (*p* < 0.001; Figure 4(a)) and increased for the VL in SUP20 (*p* = 0.021; Figure 4(b)) comparing baseline and post-NMES. There was also an interaction of *position* by *time* (*F*_3,57_ = 9.46, *p* < 0.001, *η*_*ρ*_^2^: 0.25, power: 0.96), showed as a surrogate of the QF median frequency by collapsing its superficial constituents (Figure 4(d)). There was also a significant increase in median frequency in SUP20 (*p* = 0.021) after QMECs compared to baseline.

## 4. Discussion

We demonstrated that NMES-induced contraction fatigability depends on QF muscle length according to hip and knee joint angle manipulation. Our major new findings were as follows: (i) after NMES, all positions except SUP20 had a reduction in MVC, compared to baseline; (ii) only positions with the knee at 60° of knee flexion were able to generate fatigue during NMES, which was significant from the 5^th^ (SUP60) and 7^th^ (SIT60) QMEC; (iii) fatigue was accompanied by an increase in QF nRMS and a reduction in median frequency for SUP60 and QF rRMS reduction for SUP20 and SIT20; (iv) SUP20, the only position without reduction in MVC, had an increase in the median frequency, mainly contributed by the VL. Our findings may help clinicians interpret contraction fatigability onset in their protocols of NMES in an attempt to design more rational clinical stimulation strategies.

### 4.1. Fatigue during Quadriceps Maximal Evoked Contractions

Contraction fatigability during NMES was observed only in the positions with the knee at 60° of flexion. These positions (SUP60 and SIT60) also had greater absolute QMEC than SUP20 and SIT20 (Figure 1). Similarly, a previous study reported greater fatigue at the joint angles in which the muscle generated greater force in pre fatigue state (greater torque at 65° compared to 20° and 90°) [12]. Other studies with electric stimulation also support these findings, adding the rationale for the mechanisms underlying greater fatigability, like increased metabolic rate and excitation-contraction coupling impairment [13], showing greater peripheral fatigue of the vastus intermedius [30] and muscle damage [31]. However, some studies showed greater fatigue at shorter muscle lengths [32, 33]. Finally, a recent study demonstrated that voluntary contraction with an extended knee angle (30°) was more resistant to fatigue than 60° and 90° due to decreased oxygen consumption at 30° [10]. Further mechanistic studies are necessary to elucidate this topic during NMES-induced fatigue protocols.

In the fresh state, we demonstrated that a hip extended position (SUP60) generated greater evoked torque than a position with the hip flexed (SIT60), in turn promoting greater and earlier fatigue. To the best of our knowledge, this is the first study to manipulate QF length on the hip angle during NMES for fatigue assessment. Previous studies [14, 15] found that a lying position could generate a greater evoked torque compared to seated (for a knee flexion angle of 90°), but contraction fatigability was not assessed. In the present study, faster fatigue onset in the SUP60 may indicate a greater mechanical load imposed on the QF associated with improved force generation on the elongated RF [34]. However, other mechanisms could be involved, including changes in compliance on the force transmission components of the knee extensor mechanism [35] and intermuscular connections between the QF' constituents [22].

### 4.2. Contraction Fatigability after Neuromuscular Electrical Stimulation

For the MVC obtained in baseline and post-NMES (Figure 2(a)), torque reduction was detectable in most conditions (SUP60, SIT60, and SIT20), except SUP20 condition. Interestingly, fatigue had not been settled in SIT20 during QMECs, but it was showed right after in the MVC. Currently, the onset mechanism (central or peripheral) underlying NMES-induced contraction fatigability is not well fully established, which would require electrophysiologic results like the M-wave amplitude. To date, it is known that voluntary isometric contractions generate central fatigue first, then peripheral fatigue [19], which could also be the case for QMECs, causing a reduction in voluntary torque without evoked torque changes for SIT20. However, care must be taken with this interpretation because torque level during NMES is significantly lower than that produced during MVC. Thus, even during QMEC, the low torques may hide the instant where maximal force generation was reduced.

In SUP20, the elongation of the RF at the hip was responsible for nulling the onset of fatigue in our protocol, which may be explained by the increase in median frequency, as presented in the following session. Thus, we suggest that QF performance changes could be expected through hip angle variations. Despite the RF being the only biarticular constituent of the QF, all constituents share the same insertion and major peripheral nerve (i.e., the femoral nerve) [36]. The synergistic muscles share intermuscular connective tissues that allow an anatomical and mechanical interdependency [22]. Furthermore, concerns about greater sensory discomfort during maximum contractions in shortened muscle lengths (in the case of SIT20) have been described by some authors [2]. This could explain different responses obtained in SUP20 and SIT20. These hypotheses are speculative, and more studies are needed to understand this complex outcome.

The contraction fatigability index showed greater torque reduction for SIT20 than SUP60 and SIT60. Possibly, this happened due to the lower baseline torque values of SIT20, making the percentage reduction greater than in the other positions with 60° of knee flexion. Indeed, a recent study with voluntary contraction [10] demonstrated that a more extended knee angle (30°) was more resistant to fatigue than 60° and 90° due to decreased oxygen consumption at 30°. Torque generation is related to the improved transmission of the muscle force to the tendon and optimal sarcomere/fiber length, which are critical factors responsible by physiologic architectural configuration for force generation improvements [37]. Thus, in clinical practice, it is essential to emphasize that higher torque and current NMES-efficiency accompanied by lower perceived discomfort are relevant strategies to improve strengthening and movement patterns.

### 4.3. nRMS and Median Frequency

In SUP60 (Figures 3(c)–3(e)), after QMEC, all QF constituents contributed to a small increment in the RMS despite a reduction in MVC (Figure 2(a)), which resulted in greater nRMS in this position (Figure 3(b)). The increase in nRMS on the fatigue onset was previously demonstrated as an attempt to increase motor unit recruitment [18]. In the current study, the failure to maintain the MVC torque level occurred despite this increased motor unit recruitment, suggesting peripheral fatigue [38]. In SIT60, the rRMS tended to be reduced (except for the VM), accompanying the reduction in MVC. Thus, the nRMS remained unchanged. The positions with the knee at 20° of flexion demonstrated a greater RMS/torque ratio in the fresh and fatigued states, indicating a compensatory mechanism to generate more force [39]. This effect can be related to actin-myosin complex mismatch, as expected in shortened positions. Consequently, this fact probably precipitated the activation deficit with fatigue, demonstrated by the consistent rRMS reduction.

In SUP60, there was a reduction in the median frequency of RF, which was previously found after fatiguing voluntary isometric contractions for the knee [19] and elbow extensors [18]. Thus, in fatigued states, not increasing the MF, i.e., the rate of alpha motor neuron discharge by the central nervous system [40], maybe an important factor in reducing force generation capacity. The RF may be key in the slightly greater evoked torque observed on SUP60 than SIT60 (Figure 1). Interestingly, in SUP60, only RF showed a reduction in MF (Figure 4(a)). In SUP20, the only position that did not manifest a reduction in MVC, we found an increase in the median frequency (Figures 3(b) and 3(d)). For this position, VL was the main responsible for this compensatory increase in the power spectrum, which may indicate either a shift in the type of the motor unit recruited or motor unit firing rate, which are essential factors for muscle fatigue recovery [41]. Additionally, the median frequency tended to gradually increase from the most elongated (SUP60) to the most shortened (SIT20) condition, which was previously demonstrated [42, 43].

### 4.4. Limitations

Some limitations in the present study must be highlighted. This study is part of a broader study that required torque reliability for QMEC. Thus, we allowed a rest period of two minutes between contractions. Moreover, we gradually incremented the current amplitude after each contraction, when allowed by the volunteer, to compensate the neuromuscular accommodation to the electrical current [3] and maintain the true QMEC to a discomfort level of 8/10. Despite this, we argue that this strategy is realistic because it is recommended in clinical practice [3] and allows us to detect only fatigue-related changes in the QF (not only an accommodation to the electrical current). Moreover, there are also other tools for contraction fatigability assessment that we did not use (e.g., M-wave amplitude, metabolic pathways), and we did not consider the EMG contribution of the deep vastus intermedius. Finally, our results are limited to our specific angles, population, and time frame. Thus, whether longer periods of change hip and knee joint angles will continue to determine contraction fatigability onset remains a provocative hypothesis for further investigation.

### 4.5. Practical Implications

NMES-induced contraction fatigability may be desirable or should be postponed according to training objectives. For example, functional electrical stimulation is often used in lengthy activities, like walking [44] and cycling [45], while NMES for strengthening and hypertrophy requires overload in relatively shorter exercises [3]. In the former application, early fatigue is avoided to allow activity completion, while in the latter, fatigue will probably be indicative of high training intensity, so it should be expected. We demonstrated that muscle length modulates fatigue onset, which suggests that hip and knee joint angles may be controlled strategically according to the training purposes and specificities. Current data reinforce the utilization of angle manipulation for an evidence-based approach to clinical decisions.

## 5. Conclusions

In summary, QF NMES-induced contraction fatigability is dependent on muscle length changes by both hip and knee joint angles. Contraction fatigability is greater when the knee is flexed at 60° than 20°. When the knee is flexed at 60°, a supine position promotes earlier fatigue, but when the knee is flexed at 20°, a supine position delays fatigue onset when compared to the seated position. EMG signal analysis revealed an increase in QF RMS values and a reduction in RF median frequency in SUP60 position. In SUP20, an increase in the median frequency probably favored torque level maintenance. In SIT20, there was a reduction in MVC, but not in evoked torque. These results provide a rationale for lower limb positioning during NMES, which depends on training objectives, e.g., strengthening or task-specific functionality training.

## Figures and Tables

**Figure 1:** Quadriceps maximum evoked contraction in absolute (N.m; (a)) and relative (%; (b)) values during the 1st to the 12th contraction in the positions SUP60, SIT60, SUP20, and SIT20. Data are presented as mean and 95% CI. Abbreviations: SUP60: supine with knee flexed at 60°; SIT60: seated with knee flexed at 60°; SUP20: supine with knee flexed at 20°; SIT20: seated with knee flexed at 20°. NMES: neuromuscular electrical stimulation. Statistically significant differences: ^∗^*p* < 0.05 vs. 1st contraction; ^∗∗^*p* < 0.05 vs. 1st and 2nd contractions; ^∗∗∗^*p* < 0.05 vs. 1st, 2nd, and 3rd contractions; ^a^*p* < 0.05 vs. SUP60; ^b^*p* < 0.05 vs. SIT60.

**Figure 2:** Maximum voluntary contraction in absolute (N.m; (a)) and relative (fatigue index [%]; (b)) values pre- (baseline) and post-NMES. Data are presented as mean and 95% CI. Abbreviations: SUP60: supine with knee flexed at 60°; SIT60: seated with knee flexed at 60°; SUP20: supine with knee flexed at 20°; SIT20: seated with knee flexed at 20°. NMES: neuromuscular electrical stimulation. Statistically significant differences: ^∗^*p* < 0.05 vs. baseline; ^a^*p* < 0.05 vs. SUP60; ^b^*p* < 0.05 vs. SIT60; ^c^*p* < 0.05 vs. SUP20.

**Figure 3:** Raw and normalized root mean square (RMS) pre- (baseline) and post-NMES for quadriceps constituents individually and grouped. Data are presented as mean and 95% CI. Abbreviations: SUP60: supine with knee flexed at 60°; SIT60: seated with knee flexed at 60°; SUP20: supine with knee flexed at 20°; SIT20: seated with knee flexed at 20°. NMES: neuromuscular electrical stimulation. Statistically significant differences: ^∗^*p* < 0.05 vs. baseline; ^a^*p* < 0.05 vs. SUP60; ^b^*p* < 0.05 vs. SIT60.

**Figure 4:** Median frequency pre- (baseline) and post-NMES for quadriceps constituents individually and grouped. Data are presented as mean and 95% CI. Abbreviations: SUP60: supine with knee flexed at 60°; SIT60: seated with knee flexed at 60°; SUP20: supine with knee flexed at 20°; SIT20: seated with knee flexed at 20°. NMES: neuromuscular electrical stimulation. Statistically significant differences: ^∗^*p* < 0.05 vs. baseline.

## Data Availability

The data (software raw files and spreadsheet) could be provided under request.

## Abbreviations

NMES: Neuromuscular electrical stimulation
MVC: Maximal voluntary contraction
QMEC: Quadriceps maximum evoked contraction
QF: Quadriceps femoris
RF: Rectus femoris
VL: Vastus lateralis
VM: Vastus medialis
EMG: Electromyography or electromyographic
RMS: Root mean square
rRMS: Raw root mean square
nRMS: Normalized root mean square.

## References

[1] Knutson J. S., Fu M. J., Sheffler L. R., Chae J. (2015). Neuromuscular electrical stimulation for motor restoration in hemiplegia. *Physical Medicine and Rehabilitation Clinics of North America*.

[2] Herzig D., Maffiuletti N. A., Eser P. (2015). The application of neuromuscular electrical stimulation training in various non-neurologic patient populations: a narrative review. *PM & R : The Journal of Injury, Function, and Rehabilitation*.

[3] Maffiuletti N. A. (2010). Physiological and methodological considerations for the use of neuromuscular electrical stimulation. *European Journal of Applied Physiology*.

[4] Jubeau M., Duhamel G., Wegrzyk J. (2015). Localized metabolic and t2 changes induced by voluntary and evoked contractions. *Medicine and Science in Sports and Exercise*.

[5] Jubeau M., Sartorio A., Marinone P. G. (2008). Comparison between voluntary and stimulated contractions of the quadriceps femoris for growth hormone response and muscle damage. *Journal of Applied Physiology*.

[6] Allen D. G., Lamb G. D., Westerblad H. (2008). Skeletal muscle fatigue: cellular mechanisms. *Physiological Reviews*.

[7] Enoka R. M., Duchateau J. (2016). Translating fatigue to human performance. *Medicine and Science in Sports and Exercise*.

[8] Bastos J. A. I., Martins W. R., Júnior G. C., Collins D. F., Durigan J. L. Q. (2021). Contraction fatigue, strength adaptations, and discomfort during conventional versus wide-pulse, high-frequency, neuromuscular electrical stimulation: a systematic review. *Applied Physiology, Nutrition, and Metabolism*.

[9] Chan A. Y., Lee F. L. L., Wong P. K., Wong C. Y. M., Yeung S. S. (2001). Effects of knee joint angles and fatigue on the neuromuscular control of vastus medialis oblique and vastus lateralis muscle in humans. *European Journal of Applied Physiology*.

[10] Pethick J., Winter S. L., Burnley M. (2021). Fatigue-induced changes in knee-extensor torque complexity and muscle metabolic rate are dependent on joint angle. *European Journal of Applied Physiology*.

[11] Fitch S., McComas A. (1985). Influence of human muscle length on fatigue. *The Journal of Physiology*.

[12] Marion M. S., Wexler A. S., Hull M. L., Binder-Macleod S. A. (2009). Predicting the effect of muscle length on fatigue during electrical stimulation. *Muscle & Nerve*.

[13] Lee S. C., Braim A., Becker C. N., Prosser L. A., Tokay A. M., Binder-Macleod S. A. (2007). Diminished fatigue at reduced muscle length in human skeletal muscle. *Muscle & Nerve*.

[14] Bampouras T. M., Reeves N. D., Baltzopoulos V., Maganaris C. N. (2017). The role of agonist and antagonist muscles in explaining isometric knee extension torque variation with hip joint angle. *European Journal of Applied Physiology*.

[15] Maffiuletti N. A., Lepers R. (2003). Quadriceps femoris torque and EMG activity in seated versus supine position. *Medicine and Science in Sports and Exercise*.

[16] Wan J. J., Qin Z., Wang P. Y., Sun Y., Liu X. (2017). Muscle fatigue: general understanding and treatment. *Experimental & Molecular Medicine*.

[17] Wang L., Wang Y., Ma A. (2018). A comparative study of EMG indices in muscle fatigue evaluation based on grey relational analysis during all-out cycling exercise. *BioMed Research International*.

[18] Hussain J., Sundaraj K., Subramaniam I. D., Lam C. K. (2019). Analysis of fatigue in the three heads of the triceps brachii during isometric contractions at various effort levels. *Journal of Musculoskeletal & Neuronal Interactions*.

[19] Babault N., Desbrosses K., Fabre M. S., Michaut A., Pousson M. (2006). Neuromuscular fatigue development during maximal concentric and isometric knee extensions. *Journal of Applied Physiology*.

[20] Cifrek M., Medved V., Tonković S., Ostojić S. (2009). Surface EMG based muscle fatigue evaluation in biomechanics. *Clinical Biomechanics*.

[21] Glaviano N. R., Saliba S. (2016). Can the use of neuromuscular electrical stimulation be improved to optimize quadriceps strengthening?. *Sports Health*.

[22] Maas H., Sandercock T. G. (2010). Force transmission between synergistic skeletal muscles through connective tissue linkages. *Journal of Biomedicine & Biotechnology*.

[23] Grob K., Manestar M., Filgueira L., Kuster M. S., Gilbey H., Ackland T. (2018). The interaction between the vastus medialis and vastus intermedius and its influence on the extensor apparatus of the knee joint. *Knee Surgery, Sports Traumatology, Arthroscopy*.

[24] Pincivero D. M., Salfetnikov Y., Campy R. M., Coelho A. J. (2004). Angle- and gender-specific quadriceps femoris muscle recruitment and knee extensor torque. *Journal of Biomechanics*.

[25] Fitzgerald G. K., Piva S. R., Irrgang J. J. (2003). A modified neuromuscular electrical stimulation protocol for quadriceps strength training following anterior cruciate ligament reconstruction. *The Journal of Orthopaedic and Sports Physical Therapy*.

[26] Bremner C. B., Holcomb W. R., Brown C. D. (2015). Knee joint angle influences neuromuscular electrical stimulation-induced torque. *Athletic Training and Sports Health Care*.

[27] Scott W., Adams C., Fisher J., Fisher S., Jones K., Mathieu B. (2021). Electrically elicited quadriceps muscle torque: comparison at three knee angles. *Physiotherapy Theory and Practice*.

[28] Cavalcante J. G. T., Marqueti R. . C., Geremia J. M. (2021). The effect of quadriceps muscle length on maximum neuromuscular electrical stimulation evoked contraction, muscle architecture, and tendon-aponeurosis stiffness. *Frontiers in Physiology*.

[29] Jeon W., Griffin L. (2018). Effects of pulse duration on muscle fatigue during electrical stimulation inducing moderate-level contraction. *Muscle & Nerve*.

[30] Ando R., Tomita A., Watanabe K., Akima H. (2018). Knee joint angle and vasti muscle electromyograms during fatiguing contractions. *Clinical Physiology and Functional Imaging*.

[31] Fouré A., Ogier A. C., Guye M., Gondin J., Bendahan D. (2020). Muscle alterations induced by electrostimulation are lower at short quadriceps femoris length. *European Journal of Applied Physiology*.

[32] Sacco P., McIntyre D. B., Jones D. A. (1994). Effects of length and stimulation frequency on fatigue of the human tibialis anterior muscle. *Journal of Applied Physiology*.

[33] Rassier D. E. (2000). The effects of length on fatigue and twitch potentiation in human skeletal muscle. *Clinical Physiology*.

[34] Herzog W., Abrahamse S. K., ter Keurs H. E. (1990). Theoretical determination of force-length relations of intact human skeletal muscles using the cross-bridge model. *Pflügers Archiv*.

[35] Raiteri B. J. (2018). Aponeurosis behaviour during muscular contraction: a narrative review. *European Journal of Sport Science*.

[36] Glenn L. L., Samojla B. G. (2002). A critical reexamination of the morphology, neurovasculature, and fiber architecture of knee extensor muscles in animal models and humans. *Biological Research for Nursing*.

[37] Lieber R. L., Friden J. (2000). Functional and clinical significance of skeletal muscle architecture. *Muscle & Nerve*.

[38] Harnie J., Cattagni T., Cornu C., McNair P., Jubeau M. (2020). Acute effect of tendon vibration applied during isometric contraction at two knee angles on maximal knee extension force production. *PLoS One*.

[39] Suydam S. M., Buchanan T. S., Manal K., Silbernagel K. G. (2015). Compensatory muscle activation caused by tendon lengthening post-Achilles tendon rupture. *Knee Surgery, Sports Traumatology, Arthroscopy*.

[40] Allison G. T., Fujiwara T. (2002). The relationship between EMG median frequency and low frequency band amplitude changes at different levels of muscle capacity. *Clinical Biomechanics*.

[41] Farina D., Fosci M., Merletti R. (2002). Motor unit recruitment strategies investigated by surface EMG variables. *Journal of Applied Physiology*.

[42] Farina D., Merletti R., Nazzaro M., Caruso I. (2001). Effect of joint angle on EMG variables in leg and thigh muscles. *IEEE Engineering in Medicine and Biology Magazine*.

[43] Potvin J. R., Bent L. R. (1997). A validation of techniques using surface EMG signals from dynamic contractions to quantify muscle fatigue during repetitive tasks. *Journal of Electromyography and Kinesiology*.

[44] Tenniglo M. J. B., Buurke J. H., Prinsen E. C., Kottink A. I. R., Nene A. V., Rietman J. S. (2018). Influence of functional electrical stimulation of the hamstrings on knee kinematics in stroke survivors walking with stiff knee gait. *Journal of Rehabilitation Medicine*.

[45] Allen B. C., Stubbs K. J., Dixon W. E. (2020). Characterization of the time-varying nature of electromechanical delay during FES-cycling. *IEEE Transactions on Neural Systems and Rehabilitation Engineering*.

